RETRACTED

# Arsenic in the Food Chain in Pakistan: Assessing Risks to Human Health and Ensuring Food Security Through Comprehensive Contamination Mitigation Strategies

**DOI:** 10.7759/cureus.54069

**Published:** 2024-02-12

**Authors:** Syed Shameel Ahmed Quadri, Rabia Ali, Anderson Mesidor, Imam Ali Shah, Nimra Raqeeb, Muhammad Omer Afzal, Muhammad Rizwan, Tariq Rafique, Saba Nosheen

**Affiliations:** 1 Political Science, University of Karachi, Karachi, PAK; 2 General Practice, SHED Foundation Hospital, Karachi, PAK; 3 Medical Education, Université d'État d'Haïti, Port-au-Prince, HTI; 4 Internal Medicine, Chandka Medical College, Shaheed Mohtarma Benazir Bhutto Medical University, Larkana, PAK; 5 Zoology, Mirpur University of Science and Technology, Mirpur, PAK; 6 Center for Agricultural Biochemistry and Biotechnology, University of Agriculture Faisalabad, Faisalabad, PAK; 7 School of Energy Science and Engineering, Central South University, Changsha, CHN; 8 Medical Affairs, Dadabhoy Institute of Higher Education, Karachi, PAK; 9 Editorial Board, Research Journal of Innovative Ideas and Thoughts, Faisalabad, PAK

**Keywords:** hyperkeratosis, skin disorders, cancers, health risks, arsenic toxicity, soil contamination, human health, food chain, environmental pollution, arsenic

## Abstract

Arsenic is a natural element found in the earth’s crust and is extensively present in various environmental components. Anthropogenic activities and a few natural events have generated contaminants that have led to massive environmental pollution, one form of which is arsenic contamination. Arsenic enters the human food chain via contaminated crops, water, seafood, and dairy products. In Pakistan, the increasing concentration of arsenic in the water is causing major health problems. Due to the serious health risks posed by arsenic, it is crucial to design and implement strategies for reducing and preventing the bioaccumulation of arsenic and its entry into the human food chain. There is a need for an institutional framework for arsenic mitigation, accountability, and systemic checks and balances. Targeted short- and long-term policies are required for effective and sustainable management.

## Introduction and background

Human development is majorly attributed to industrialization and urbanization. However, anthropogenic activities and a few natural events have led to massive environmental pollution. Arsenic (As) is a natural element in the earth’s crust. It is extensively present in various environmental components. The atomic weight, specific gravity, boiling point, and melting point of arsenic are 74.9 g/mol, 5.73 g cm^-3^, 614°C, and 817°C, respectively. It has a silver-gray color and occurs in a firm crystalline form. It has high industrial value and is used to manufacture semiconductors, pesticides, herbicides, fertilizers, cosmetics, paints, glass, ammunition, fireworks, etc. Such a wide range of use renders an arsenic-free environment challenging [1].

RETRACTED

According to the International Agency for Research on Cancer, inorganic arsenic is classified as a group 1 carcinogen [2], and according to the Agency for Toxic Substances and Disease Registry, it is considered embryotoxic, genotoxic, and neurotoxic [3]. Soil health affects plant growth and productivity, and it is linked to human health and food security. Soil-bound arsenic can be transferred to plant parts that humans consume. Prolonged consumption of contaminated crops poses serious health hazards for humans [4]. Arsenic also enters the food chain by consuming contaminated water, seafood, and dairy products. Food products such as milk, eggs, fish, meat, poultry, and dairy are derived from animal sources. They can be contaminated if animals consume arsenic-contaminated water and crops or thrive in a contaminated environment [5]. The study will emphasize contamination of the food chain and resulting health hazards and disorders because of arsenic toxicity. Moreover, the study will highlight the strategies for mitigating arsenic contamination.

The research conducted in Pakistan since the beginning of the twenty-first century is incorporated into this study. The study particularly focuses on regions that are experiencing difficulties with arsenic poisoning. Attention was paid to peer-reviewed articles and scientific studies that offered concrete proof of arsenic pollution. Individuals at a greater risk of being exposed to arsenic were the subjects of the primary geographical focus of concern. The human populations of interest for this study were those situated in areas with a significant concern over arsenic contamination in water, soil, and agricultural products. In addition, studies that did not include any empirical data or evaluations of treatments were not considered for inclusion in the review. Regarding language, any study not available in the English language was not considered for inclusion as there may be limitations in the resources available for translation.

## Review

Bioaccumulation of arsenic in Pakistan

Contamination of water with arsenic is a global concern. In Pakistan, the increasing concentration of arsenic in water is causing major health problems, as mentioned in Table 1. Populations of Sindh and Punjab are particularly at risk of arsenic contamination in water. According to estimates, about 36% of the population in Sindh is facing the risk of arsenic toxicity as the level of arsenic in drinking water is above the safe threshold of 10 mg/L [6]. In Punjab, 20-30% of water resources have arsenic contamination above the safe threshold [7,8]. In a national survey conducted in 2001 in which water samples from 35 districts were analyzed, the findings were alarming. The survey showed that 70% of samples contained higher arsenic levels than those deemed safe by the World Health Organization, with 9% of samples having arsenic concentrations >10 mg/L [9]. This elevated concentration was due to water contamination from pesticides, industrial activities, and other anthropogenic causes. Another survey was conducted to analyze arsenic concentrations in underground water in Rahim Yar Khan district in Punjab. Results showed that arsenic concentration ranged from 150 to 400 µg/L. Crops such as sugarcane and cotton are cultivated in this area. Thus, high amounts of pesticides and fertilizers are released into the water [10]. Studies suggest that the presence of phosphatic fertilizers in the soil increases the concentration of arsenic [11], with the Pakistan Council of Research in Water Resources confirming raised phosphate concentrations in the district.

RETRACTED

**Table 1:** Arsenic contamination in water in Pakistan.

Location	Population at risk	Arsenic level (mg/L)	Reference
Sindh	36%	Above 10	[6]
Punjab	20–30%	Above 10	[7,8]
National survey	70% samples	Above the WHO threshold	[9]
Rahim Yar Khan	Not specified	150–400	[10]

Arsenic is present in soil and subsoil surfaces in Pakistan, as mentioned in Table 2, with deep soils having higher concentrations than surface soil in the same region. Agricultural areas of Sindh had the highest soil concentration of 46.1 mg/kg [12], followed by 36 mg/kg in the soil from different areas of Punjab [13]. It was found that fertilizers and air pollutants due to coal burning caused higher arsenic concentrations in topsoil. The United States Environmental Protection Agency found that in some regions of Sindh, the total arsenic concentration in soils and sediments was higher than the safe threshold [14]. Arsenic concentration in Manchar Lake sediments ranged from 11.2 to 55.4 mg/kg [12]. Toxic ions either remain on the soil surface or leach into groundwater. This enters the food chain and contaminates drinking water and food, accumulating in plants and humans. Staple food, vegetables, and cereals are the primary sources of entry of toxic metals into the food chain [15]. Studies show that the flow of arsenic in plants is through passive water flow. Cultivating crops in arsenic-rich land and water affects the height and yield of crops. In Sindh, accumulation of arsenic in spinach, mint, and coriander leaves ranged from 0.91 to 1.21 mg/kg, while arsenic uptake in potato, carrot, and onion ranged from 0.048 to 0.256 mg/kg, as mentioned in Table 3. The daily intake of arsenic through food in arsenic-endemic regions was 343.5 g/day, while in the unaffected region was 144.7 g/day [12]. Thus, communities in such regions are highly exposed to the harmful impacts of arsenic toxicity through food, water, or animal-based products. It is essential to address this issue as a matter of immediate concern.

RETRACTED

**Table 2:** Arsenic in soil in Pakistan.

Region	Soil arsenic concentration (mg/kg)	Source
Agricultural areas	46.1	Highest in Sindh [12]
Different areas of Punjab	36	[13]
Manchar Lake sediments	11.2–55.4	[12]

**Table 3:** Arsenic accumulation in crops and daily intake.

Crop	Arsenic concentration (mg/kg)	Daily intake (g/day)	Region	Reference
Spinach, mint, and coriander	0.91–1.21	343.5 (endemic), 144.7 (unaffected)	Sindh	[12]
Potato, carrot, and onion	0.048–0.256		Sindh	[12]

Health hazards of arsenic contamination

In Pakistan, a plethora of research has been conducted on the health risks caused by arsenic in food. A study reported an average daily intake of 9-13 µg/kg/day of arsenic in food in rural and urban areas of Sindh and Punjab [12]. Another study reported that the hazard quotient (HQ) of arsenic in Punjab was 86% above the safe HQ (1.00) [16]. In Sindh, the HQ of arsenic concentration in the milk of goats, sheep, and cattle was also above the safe HQ value [5]. Contaminated milk can cause life-threatening diseases in children, including skin, lung, and gallbladder cancer [17]. The concentration of arsenic in cattle milk in Pakistan was higher than that in India, West Bengal, Japan, the United Kingdom, Australia, and Canada [18].

Arsenic has wide-ranging effects, including cardiovascular and neurological; however, its impact on the reproductive system has been relatively ignored. Arsenic in the uterus results in developmental abnormalities in the fetus. Epidemiological studies found that increased arsenic concentration was associated with infant mortality, congenital body defects, and decreased birth weight [19,20]. These health concerns are imminent in areas with chronic arsenic exposure. Arsenic also affects the male endocrine system. An experimental study on male rates showed that arsenic exposure caused steroidogenic dysfunction and infertility [21]. Humans may also develop this dysfunction; however, there are limited studies on the association of arsenic toxicity with male endocrine dysfunction. Research conducted on goats in Pakistan showed that in vitro sodium arsenite inhibited steroid synthesis and semen quality, leading to infertility in goats [22]. Another study reported a similar type of infertility in other regions of Pakistan exposed to increased arsenic concentration [23]. Arsenic contamination not only affects humans and animals but also plants. Arsenic in soil translocates in the root system and aerial parts of plants and interferes with plant metabolism. A study found that arsenic concentration in Punjab affected seed germination and growth of wheat crops [24]. Consuming crops contaminated with arsenic causes health risks for humans and animals, as mentioned in Table 4. There is ample evidence of arsenic contamination in Pakistan’s food chain and its health effects.

RETRACTED

**Table 4:** Health risks and impact of arsenic in Pakistan.

Aspect	Details/Statistics	Reference
Daily arsenic intake in food	9–13 µg/kg/day in the rural and urban areas of Sindh and Punjab	[12]
Hazard quotient (HQ) of arsenic in Punjab	86% above the safe HQ (1.00)	[16]
Arsenic concentration in cattle milk in Pakistan	Higher than India, West Bengal, Japan, the United Kingdom, Australia, and Canada	[18]
Impact on the reproductive system	Developmental abnormalities in the fetus; associated with infant mortality, congenital defects, and decreased birth weight	[19,20]
Impact on the male endocrine system	Steroidogenic dysfunction and infertility in male rats	[21]
Arsenic in goats in Pakistan	In vitro sodium arsenite inhibits steroid synthesis and semen quality, leading to infertility	[22]
Arsenic in soil affects plant growth	Interferes with seed germination and growth of wheat crops	[24]

Strategies to mitigate arsenic contamination

About two decades ago, the United Nations International Children’s Emergency Fund (UNICEF) investigated and identified that arsenic contamination is a significant health concern in Pakistan. Unfortunately, no systemic action has been taken since then despite millions of people being at risk of severe adverse effects. Due to the serious health risks posed by arsenic, it is crucial to design and implement strategies for reducing and preventing the bioaccumulation of arsenic and its entry into the human food chain. Pakistan can learn from the successes and drawbacks of the arsenic mitigation strategy of Bangladesh. The most crucial step in the right direction will be political commitment. Policymakers and the government must demonstrate commitment to food security and protecting people from arsenic toxicity. Although the National Action Plan for Arsenic Mitigation was made following the initial survey, efforts lasted for a few years, and, ultimately, nothing was done. Low-income countries like Pakistan rely on donor aid for development and health-related projects, but this developmental model is unsustainable [25]. For instance, donors provided funds for sono filters in Bangladesh; however, prior needs assessment was not adequately done, and stakeholders were not fully involved because the project was unsuccessful [26]. UNICEF provided technical and financial support to private and government institutions in Pakistan. However, soon after the support and aid were withdrawn, actions for arsenic mitigation ended. The government should not rely on foreign aid alone, and arsenic mitigation strategies should be made a part of the budget. This will enhance local capacity and sustainability. There is a need for an institutional framework for arsenic mitigation, accountability, and systemic checks and balances [27]. Cultural and human factors such as community readiness, knowledge, support, engagement, participation acceptance, and resources can challenge the sustainability of any program. These factors should be taken into account while developing a mitigation plan. Targeted short- and long-term policies are required for effective management. Some of the policy recommendations and strategies for contamination mitigation are presented below.

RETRACTED

Short-term interventions

The population at the highest risk should be emphasized in the short term. Such communities should have immediate, affordable, acceptable arsenic removal technology, surface treatment, and deep wells.

Arsenic Removal Technology

Technology selection should be based on its operation and maintenance requirements, long-term sustainability, socioeconomic status of the population, and networking of stakeholders. The Pakistan Council of Research in Water Resources has developed arsenic removal technologies, and similar strategies have been effectively implemented in Bangladesh and India. Pakistan can modify and adopt these strategies. Techniques such as membrane purification and ion exchange are costly, hi-tech, and require extensive training. Thus, these are not suitable in Pakistan. For Pakistan, methods such as precipitation and oxidation are better suited [28].

Coagulation and Flocculation

This method includes co-precipitation and coagulation. It is simple and cost-effective and uses local materials such as iron chloride, iron sulfate, and alum. However, it is inefficient and requires pre-oxidation [29].

Jerry Can Technique

This method involves adsorption and precipitation. It can yield 73,000 L of water. It is cost-effective and can be set up in rural areas [28].

Bottom Ash System

It is an arsenic removal system that operates on coal ash. Coal ash is readily available from combustion units and coal power plants. It has a low initial cost, yields 73,000 L, and is suitable for rural communities.

RETRACTED

Solar Distillation

In this method, sunlight is used for water evaporation and condensation. It is a cheap and eco-friendly technology for the decontamination of water [30].

Kanchan Filters

This system uses iron nails, sand, brick chips, and gravel. It is a cheap option and can be implemented at the household level. It has a high water filtration rate and yields 80,000 L [31].

Long-term interventions

Effective risk reduction is possible with practical long-term policy and implementation which requires planning, technical and financial resources, and commitment. Long-term strategies for mitigating arsenic contamination in the food chain are discussed below.

Genetic Engineering

Genetic manipulation includes different strategies depending upon the goal, such as increased tolerance for arsenic-contaminated environment, decreased uptake of arsenic in crop plants, or increased methylation. It is difficult to entirely block the entry of arsenic in crop plants because a single transport system in plants is used for beneficial or essential elements. Nevertheless, increased production of phytochelatin in roots can restrict the translocation of arsenic in edible plants through arsenic-phytochelatin complexes and vacuolar sequestration. Genetic manipulation can also convert toxic arsenic species into volatilizable or methylated forms [31].

Piped Water Supply

Pipe water supply to the domestic population should be from arsenic-free reservoirs. The government should develop infrastructure and allocate resources to ensure the long-term protection of vulnerable communities. The supply can be in standposts, yard connections, or house connections, depending on the affordability and availability of resources [31].

Micro Watershed System

This system can be used for storing rainwater, which can be treated and used in households. It requires surveys to identify storage locations depending on rain patterns. Due to varying weather throughout the year and periods of dry spells, a large storage capacity is required for continuous water supply to the communities.

Soil Investigation

The quality of soil and subsoil surface should be investigated routinely as the arsenic content in soil is transferred to edible crop plants and water. The data can be used for future planning of agriculture and water infrastructure.

The short- and long-term interventions for mitigating arsenic contamination in the food chain are summarized in Table 5.

**Table 5:** Strategies to mitigate arsenic contamination.

Intervention	Details/Description	Reference
Arsenic removal technology	Selection based on operation and maintenance, sustainability, socioeconomic status, and stakeholder networking; The Pakistan Council of Research in Water Resources technologies can be adopted	[28]
Coagulation and flocculation	Simple and cost-effective operation using local materials such as iron chloride, iron sulfate, and alum; requires pre-oxidation	[29]
Jerry can technique	Involves adsorption and precipitation; yields 73,000 L; cost-effective for rural areas	[28]
Bottom ash system	An arsenic removal system operating on coal ash; low initial cost, yields 73,000 L; suitable for rural communities	[28]
Solar distillation	Utilizes sunlight for water evaporation and condensation; cheap and eco-friendly	[30]
Kanchan filters	Uses iron nails, sand, brick chips, and gravel; a cheap option suitable for household-level implementation; high water filtration rate, yields 80,000 L	[31]
Genetic engineering	Strategies for increased tolerance, decreased uptake, or increased methylation of arsenic in crop plants; production of phytochelatin in roots restricts the translocation of arsenic	[31]
Piped water supply	Arsenic-free reservoirs supplying the domestic population through stand posts, yard connections, or house connections; requires infrastructure development and resource allocation	[31]

RETRACTED

## Conclusions

Contamination of food crops, soil, and water resources due to geological and anthropogenic sources is a profound health concern. The literature highlights threats and health defects caused by arsenic toxicity in the food chain, mainly vegetables and grains. Given the evidence of arsenic in animal secretions, livestock-based food products significantly contribute to contamination, particularly in areas where fertilizers and pesticides are abundantly used. Chronic exposure leads to cancers and respiratory, reproductive, developmental, endocrinological, neurological, and skin diseases. It is a significant health concern and needs preventive strategies to minimize risks. There is a dire need for a national action plan for mitigating arsenic contamination. For sustainable outcomes, mitigating interventions should be conjugated with political commitment and social mobilization.
